# Dexmedetomidine protects H9C2 rat cardiomyocytes against hypoxia/reoxygenation injury by regulating the long non-coding RNA colon cancer-associated transcript 1/microRNA-8063/Wnt/β-catenin axis

This article has been retracted.

**DOI:** 10.1080/21655979.2022.2080420

**Published:** 2022-05-29

**Authors:** Chundong Liu, Rui Xu

**Affiliations:** Department of Anesthesiology, Wuhan Fourth Hospital, Wuhan, Hubei, China

**Keywords:** Dex, H9C2, H/R, lncRNA CCAT1, miR-8063

## Abstract

Dexmedetomidine (Dex) protects the heart from ischemia/reperfusion (I/R) injury. The differential expression of long non-coding RNAs (lncRNAs) is associated with myocardial injury, but whether the lncRNA colon cancer-associated transcript 1 (CCAT1) is associated with Dex-mediated myocardial protection remains unclear. In this study, a hypoxia/reoxygenation (H/R) H9C2 model was established to simulate the in vitro characteristics of I/R. CCAT1 and microRNA (miR)-8063 expression levels in H/R H9C2 cells pretreated with Dex were determined via quantitative reverse transcription-polymerase chain reaction. The survival and apoptotic rates of H9C2 cells were determined via cell counting kit-8 and flow cytometry assays. Wnt3a, Wnt5a, and β-catenin protein levels were measured via western blotting. Luciferase and RNA immunoprecipitation assays were used to explore the binding relationship between miR-8063 and CCAT1. Dex pretreatment increased H/R H9C2 cell viability and CCAT1 expression, while decreasing the cell apoptosis and Wnt3a, Wnt5a, and β-catenin protein levels. Knockdown of CCAT1 abolished the protective effects of Dex on H/R H9C2 cells, and the downregulation of miR-8063 expression eliminated the effect of CCAT1 knockdown. These results revealed that CCAT1, a sponge for miR-8063, is involved in Dex-mediated H9C2 cell H/R injury by negatively targeting miR-8063 and inactivating the Wnt/β-catenin pathway. Dex protects H9C2 cells from H/R impairment by regulating the lncRNA CCAT1/miR-8063/Wnt/β-catenin axis.

## Highlights

- H/R induces the downregulation of CCAT1 and upregulation of miR-8063 levels in H9C2 cells.
- Dex increases H/R H9C2 cell viability and decreases apoptosis via the Wnt/β-catenin pathway.
- miR-8063 inhibitor eliminates the effects of CCAT1 knockdown on H/R H9C2 cells treated with Dex.
- CCAT1 sponges miR-8063 in H9C2 cells.

## Introduction

Myocardial infarction (MI) involves the oxidative damage and apoptosis of cardiomyocytes resulting from the pathological ischemia of the heart [1]. Currently, the standard treatment for MI is timely restoration of ischemic myocardial blood flow (reperfusion), which enhances the long-term myocardial function, limits the infarct size, alters the infarct healing patterns, and reduces the mortality of patients [2]. However, there is considerable experimental and clinical evidence that reperfusion can cause additional myocardial/reperfusion injury, which is a major cause for chronic heart failure [3,4]. Hence, reducing the inevitable ischemia/reperfusion (I/R) damage during ischemia and reperfusion remains a challenge in cardiac therapy [5].

Cellular hypoxia/reoxygenation (H/R) is often used to simulate the in vitro characteristics of I/R to investigate the impact of cardioprotective strategies on myocardial damage [6,7]. Cell viability decreases and apoptosis increases after H/R-induced cell impairment [8].

Dexmedetomidine (Dex) is an extremely selective α2-adrenergic receptor agonist that is utilized for anti-salivation, analgesia, and sedation, and exerts therapeutic effects during cardiac dysfunction [9,10]. Dex alleviates H/R-induced myocardial cell injury. For example, Zhu et al. [11] found that 1 µM Dex could attenuate H9C2 cardiomyocyte injury by inhibiting endoplasmic reticulum stress. Yin et al. [12] showed that Dex relieves hydrogen peroxide-induced oxidative stress and cell necrosis by activating α2-adrenergic receptors in H9C2 cells.

Long non-coding RNAs (lncRNAs), the most common and functionally diverse ncRNAs, do not encode protein information and are > 200 nucleotides in length [13]. The lncRNA colon cancer-associated transcript 1 (CCAT1), a widely studied lncRNA, acts as an oncogene in various tumors [14]. CCAT1 is suggested to promote tumor progression by promoting the proliferation of cancer cells and inhibiting their apoptosis [15]. In cell-damaging diseases, such as preeclampsia, CCAT1 interferes with disease progression by increasing trophoblast proliferation and accelerating the cell cycle [16]. Therefore, CCAT1 exerts different effects in different types of diseases. A study on hepatocyte oxygen glucose deprivation/reperfusion (OGD/R) revealed that CCAT1 plays a protective role in OGD/R hepatocytes, and this protective effect may be achieved by synergistic Dex treatment [17]. However, the effects of CCAT1 on H/R in cardiomyocytes have rarely been reported.

In this study, we hypothesized that CCAT1 regulation may reduce H/R-induced H9C2 cell viability and abnormal apoptosis. We used the H/R model to clarify the downstream mechanism of Dex in alleviating H/R damage in H9C2 cells and explore the relationship between Dex and the CCAT1/miR-8063/Wnt/β-catenin pathway.

## Methods

### Cell culture

Immortalized rat cardiomyocytes (H9C2) were purchased from the American Type Culture Collection (USA), seeded into a 48-well plate with 2 × 10^4^ cells/well, and maintained in Dulbecco’s modified Eagle’s medium (DMEM, Gibco, USA) containing 10% fetal bovine serum (FBS) and 1% penicillin-streptomycin. The cells were cultured at 37°C and 5% CO_2_ in an atmosphere of 95% O_2_.

### H/R and Dex treatment

H/R was performed as previously described [18]. Briefly, the cells were placed in a medium in a normoxic environment (95% N_2_/5% CO_2_) overnight at 37°C. Subsequently, the medium was substituted with fresh DMEM containing 10% FBS and reoxygenated at 37°C for 2 h in an incubator containing 95% O_2_ and 5% CO_2_. Additionally, H9C2 cells were incubated with different concentrations of Dex (0, 1, 5, 10, and 20 μM) for 1 h to create the H/R + DEX group before the H/R protocol [19].

### Cell counting kit-8 (CCK-8) assay

The CCK-8 kit was used, according to the manufacturer’s instructions (Dojindo, USA). H9C2 cells were seeded in a 48-well plate and cultured for 24 h. After replacement with fresh medium, 10% CCK-8 was added and the cells were incubated for 3 h. Absorbance was measured at 450 nm using a microplate reader (Molecular Devices, USA) [20].

### Flow cytometry assay

This assay was performed using an Annexin V-fluorescein isothiocyanate (FITC)-propidium iodide (PI) Apoptosis Detection Kit (Beyotime, Shanghai, China). In short, the cells were collected, fixed in 70% cold ethanol, centrifuged, and incubated with 100 μL of RNase for 30 min at 37°C. Subsequently, FITC and PI were placed in the cell suspension for 30 min at 4°C in succession, and a flow cytometer (Beckman Coulter, USA) was used to measure the cell apoptosis rate [21].

### Quantitative reverse transcription-polymerase chain reaction (qRT-PCR)

RNAiso Plus (Takara, Japan) was used to collect the total RNA and the mirVana miRNA Isolation Kit (Ambion, USA) was used to extract the miRNA from cells, according to the manufacturers’ instructions. cDNA was synthesized from RNA using M-MLV reverse transcriptase (Takara), and miR-8063 expression levels were determined via stem-loop RT-PCR. Subsequently, a Stratagene MX3000P system (Agilent, USA) was used to conduct RT-PCR with the SYBR Green quantitative PCR SuperMix (Invitrogen, USA). Glyceraldehyde-3-phosphate dehydrogenase (GAPDH) or uracil 6 (U6) served as the normalization program to calculate the change in gene expression folding, and all data were analyzed using the 2^−ΔΔCt^ method [22]. All primer sequences are presented in Table 1.

**Table 1.** Primers used for the target genes

Gene	Primers
CCAT1	Forward: 5’-GCAGGCAGAAAGCCGTATCT-3’
	Reverse: 5’-TCCCAGGTCCTAGTCTGCTT-3’
miR-8064	Forward: 5’-TGCGGAGCACACTGAGCGG-3’
	Reverse: 5’-CCAGTGCAGGGTCCGAGGT-3’
U6	Forward: 5’-TGCTTCGGCAGCACATATAC-3
	Reverse: 5’-AGGGGCCATGCTAATCTTCT −3
GAPDH	Forward: 5’-ATGACTCTACCCACGGCAAG-3’
	Reverse: 5’-CTGGAAGATGGTGATGGGTT-3’

### Cell transfection

RiboBio (China) supplied specific CCAT1 small interfering oligonucleotides (si-CCAT1), negative control oligonucleotides (si-NC), CCAT1 overexpression vector (OE-CCAT1), and an empty vector. The miR-8063 inhibitor and NC inhibitor were purchased from SwitchGear Genomics (USA). H9C2 cells were treated with 75 nM oligonucleotides, 2 μg/mL overexpression vector, or 75 n M inhibitor using Lipofectamine 2000 (Invitrogen, USA), according to the manufacturer’s instructions. Subsequent experiments were conducted after transfection for 48 h.

### Luciferase assay

Full-length sequence and mutant *CCAT1* were amplified and delivered into the luciferase psiCHECK2 vector (Promega, USA). A wild-type plasmid (CCAT1-WT) with full-length sequence of CCAT1 containing a complementary sequence of miR-8063 was constructed. Additionally, a mutant CCAT1 plasmid (CCAT1-MUT) was constructed by mutating a complementary sequence with miR-8063. H9C2 cells were transfected with 1 μg reporter plasmid and 100 nM miR-8063 mimic or mimic-NC using Lipofectamine 2000. Luciferase activity was determined using a dual-luciferase reporter assay kit (Promega, USA), according to the manufacturer’s instructions [23].

### RNA Immunoprecipitation (RIP)

RIP assay was performed using the Magna RIP RNA-Binding Protein Immunoprecipitation Kit (Millipore, Billerica, MA, USA). Antibodies against IgG or Ago2 (diluted 1 : 50) were bound to magnetic beads. H9C2 cells were lysed using the RIP lysis buffer and immunoprecipitated using precipitation magnetic beads. Beads were then treated with proteinase K buffer solution for 0.5 h at 55°C. Subsequently, RNA was isolated and purified from the inputs and precipitated magnetic beads, and CCAT1 levels were determined via qRT-PCR [24].

### Western blotting

Total proteins from H9C2 cells lysed using the radioimmunoprecipitation assay buffer were quantified using a bicinchoninic acid kit (Thermo Scientific, USA). Proteins (20 µL) were loaded and subjected to gel electrophoresis on 10% sodium dodecyl sulfate-polyacrylamide gel electrophoresis and transferred onto polyvinylidene fluoride membranes. Membranes were then exposed to the blocking buffer for 1 h at room temperature and incubated with Wnt3a (ab234099, 1:500; Abcam, UK), Wnt5a (ab174963, 1:500; Abcam), β-catenin (ab32572, 1:500; Abcam), and GAPDH (ab8245, 1:1000; Abcam) antibodies with agitation at 4°C overnight. Subsequently, the membranes were incubated with secondary antibodies (ab6721, 1:2000; Abcam) for 1 h. Enhanced chemiluminescence western blotting substrate (Bio-Rad, USA) was used to detect the signals [25].

### Statistical analysis

The results are presented as the mean ± standard deviation and were analyzed using SPSS 17.0 (Chicago, USA). Student’s *t*-test was used to compare two groups, and one-way analysis of variance was used to compare multiple groups. All experiments were performed in triplicate. Statistical significance was set at P < 0.05.

## Results

In this study, we established an H9C2 H/R injury model and evaluated the effects of Dex, CCAT1, and miR-8063 on cell viability, apoptosis, and Wnt3a, Wnt5a, and β-catenin protein levels. We assumed that Dex protected H9C2 cells against H/R injury by promoting CCAT1 and inhibiting miR-8063 expression, while inactivating the Wnt/β-catenin pathway. We found that Dex pretreatment increased H/R H9C2 cell viability and CCAT1 levels, while decreasing apoptosis and the levels of miR-8063, Wnt3a, Wnt5a, and β-catenin. Notably, we found that CCAT1 sponges miR-8063 and inactivates the Wnt/β-catenin pathway.

### Dex pretreatment promotes the viability of H9C2 cells under H/R, inhibits apoptosis, and inactivates the Wnt/β-catenin pathway

H9C2 cells were treated with different concentrations of Dex (0, 1, 5, 10, and 20 μM) to select a suitable Dex concentration. The results showed that the cell viability of cells treated with 1, 5, 10, and 20 μM increased compared with that in the control cells (Figure 1(a)). To investigate the influence of Dex on the biological functions of H/R H9C2 cells, these cells were pretreated with 10 μM Dex due to highest cell viability. Cell viability in H/R or H/R + DEX groups decreased by 55 and 30%, respectively, compared with that in the control group, and that in the H/R + DEX group increased by more than 30% compared to that in the H/R group (Figure 1(b)). In addition, flow cytometry revealed that the apoptosis rate of cells treated with H/R was three times higher than that of cells treated with control, whereas the apoptosis rate achieved by H/R was partially alleviated by Dex pretreatment (Figure 1(c)). Moreover, western blotting revealed that Wnt3a, Wnt5a, and β-catenin protein levels were increased after H/R treatment, while the addition of Dex slightly decreased these levels (Figure 1(d)). These results suggest that Dex preconditioning may alleviate H/R-induced damage in H9C2 cells and inactivate the Wnt/β-catenin pathway.

**Figure 1.** Dex pretreatment promotes the viability of H9C2 cells under H/R and inhibits apoptosis and inactivate Wnt/β-catenin pathway (a). The cell viability in H9C2 treated with different concentrations of Dex (0, 1, 5, 10 and 20 μM) were assessed by CCK-8. (b). The H9C2 cell viability in control, H/R, and H/R + DEX were assessed by CCK-8. (c). FITC-PI kit was employed to assess cell apoptosis in H9C2 induced utilizing H/R or DEX. (d). Western blotting was utilized to measure Wnt3a, Wnt5a and β-catenin protein levels in H9C2 induced by H/R or DEX. CON, control; H/R, hypoxia/reoxygenation; Dex, dexmedetomidine. N = 3 for each group. *P < 0.05, **P < 0.001 vs. CON; #P < 0.05, ##P < 0.001 vs. H/R.

### CCAT1 prevents the reduction of H/R H9C2 cell injury induced by Dex treatment

Next, we explored the mechanism of action of CCAT1 in H/R-treated H9C2 cells. qRT-PCR analysis showed that CCAT1 expression levels in the H/R and H/R + DEX groups were decreased compared to those in the control group, while those in the H/R + DEX group were enhanced by about 1.5-fold compared with those in the H/R group (Figure 2(a)). Subsequently, the levels of CCAT1 in H9C2 cells were knocked down or upregulated to explore the changes in cell biological functions. Transfection with siRNA oligonucleotides or overexpression vector targeting CCAT1 decreased the CCAT1 expression by more than 75% or increased it by more than three times, indicating the CCAT1 was successfully knocked down or upregulated (Figures 2(b) and 3(a)). In addition, CCK-8 assay revealed that unlike the H/R + DEX + si-NC or H/R + DEX + empty vector group, the cell viability of the H/R + DEX + si-CCAT1 or H/R + DEX + OE-CCAT1 group decreased by approximately 20% or increased by approximately 1.4-fold (Figures 2(c) and 3(b)). Furthermore, flow cytometry analysis revealed that apoptosis level in the H/R + DEX + si-CCAT1 group was approximately 1.3 times higher than that in the H/R + DEX + si-NC group, while the apoptosis level in the H/R + DEX + OE-CCAT1 group was approximately 40% lower than that in the H/R + DEX + empty vector group (Figures 2(d) and 3(c)). Western blotting revealed that, in contrast to H/R + DEX + si-NC or H/R + DEX + empty vector group, Wnt3a, Wnt5a, and β-catenin protein levels were increased in the H/R + DEX + si-CCAT1 group and reduced in the H/R + DEX + OE-CCAT1 group (Figures 2(e) and 3(d)). These results indicate that the knockdown of CCAT1 partially reverses the therapeutic effect of DEX on H/R-treated H9C2 cells, leading to the deterioration of cell damage; however, upregulation of CCAT1 levels exerted the opposite effects.

**Figure 2.** Knockdown of CCAT1 worsens H9C2 cell damage under H/R (a). CCAT1 level of H9C2 cells among control (CON), H/R, or DEX treated were assayed by qRT-PCR. **P < 0.001 vs. CON; ##P < 0.001 vs. H/R. (b). The expression levels of CCAT1 were detected by qRT-PCR in H9C2 cells treated with si-NC or si-CCAT1. (c). The cell viability of H9C2 cells in H/R, H/R + DEX, H/R + DEX +si-NC, and H/R + DEX +si-CCAT1 groups was assessed by CCK-8. (d). Flow cytometry was employed to assess cell apoptosis of H9C2 cells in H/R, H/R + DEX, H/R + DEX +si-NC, and H/R + DEX + si-CCAT1. (e). Western blotting was utilized to measure Wnt3a, Wnt5a and β-catenin protein levels in H9C2 treated with H/R, H/R + DEX, H/R + DEX +si-NC, and H/R + DEX + si-CCAT1. H/R, hypoxia/reoxygenation; Dex, dexmedetomidine; si-CCAT1, CCAT1 siRNA; si-NC, negative control of si-CCAT1. N = 3 for each group. **P < 0.001 vs. H/R; #P < 0.05, ##P < 0.001 vs. H/R + DEX +si-NC.

**Figure 3.** Up-regulation of CCAT1 promotes the reduction of H/R H9C2 cell injury induced by Dex treatment (a). The expression levels of CCAT1 were detected by qRT-PCR in H9C2 cells treated with empty vector or OE-CCAT1. (b). The cell viability of H9C2 cells in H/R, H/R + DEX, H/R + DEX + empty vector, and H/R + DEX + OE-CCAT1 groups was assessed by CCK-8. (c). Flow cytometry was employed to assess cell apoptosis of H9C2 cells in H/R, H/R + DEX, H/R + DEX + empty vector, and H/R + DEX + OE-CCAT1. (d). Western blotting was utilized to measure Wnt3a, Wnt5a and β-catenin protein levels in H9C2 treated with H/R, H/R + DEX, H/R + DEX + empty vector, and H/R + DEX + OE-CCAT1. CON, control; H/R, hypoxia/reoxygenation; Dex, dexmedetomidine; si-CCAT1, CCAT1 siRNA; si-NC, negative control of si-CCAT1. N = 3 for each group. **P < 0.001 vs. H/R; #P < 0.05, ##P < 0.001 vs. H/R + DEX + empty vector.

### CCAT1 sponges miR-8063

In addition, we focused on the downstream mechanisms of CCAT1 in H9C2 cells. As illustrated in Figure 4(a), CCAT1 binds to miR-8063. Luciferase activity analysis showed that, compared to the CCAT1-WT + mimic-NC group, the luciferase activity of CCAT1-WT + miR-8063 mimic group was decreased by approximately 50% (Figure 4(b)). In addition, RIP assay revealed that CCAT1 was enriched in the miR-8063 + Ago2 group (Figure 4(c)). This confirms that CCAT1 sponges miR-8063. Additionally, changes in miR-8063 expression levels were detected in the cells. H/R treatment increased the miR-8063 levels by 2.6 times, and H/R combined with Dex increased the levels of miR-8063 by 1.5 times contrast to the control group, while the miR-8063 levels were decreased by 40% in the H/R + Dex group, in contrast to the H/R group (Figure 4(d)). In other words, the levels of miR-8063 sponged by CCAT1 were upregulated in H/R H9C2 cells.

**Figure 4.** CCAT1 sponges miR-8063 (a). The predicted target sequences in CCAT1 which can directly bind with miR-8063. (b). Luciferase reporter assay was performed to indicate that miR-8063 could directly bind with CCAT1. **P < 0.001 vs. CCAT1-WT+miR-8063 mimic. (c). RIP assay was utilized to indicate the targeting relationship between CCAT1 and miR-8063. **P < 0.001 vs. IgG. (d). miR-8063 level of H9C2 cells among control (CON), H/R, or DEX treated were assayed by qRT-PCR. H/R, hypoxia/reoxygenation; Dex, dexmedetomidine. N = 3 for each group. **P < 0.001 vs. CON; ##P < 0.001 vs. H/R.

### Interfering miR-8063 reverses the effects of CCAT1 knockdown on the behavior and the Wnt/β-catenin pathway of H/R H9C2 cells

To elucidate the effect of miR-8063 combined with CCAT1 on the biological behavior of H/R-treated H9C2 cells, miR-8063 and CCAT1 were silenced in H9C2 cells. qRT-PCR manifested that the miR-8063 levels increased by 3-fold after CCAT1 silencing and decreased by 80% after miR-8063 interference, which reversed the effects of CCAT1 silencing on miR-8063 (Figure 5(a)). In addition, CCK-8 and flow cytometry analyses showed that miR-8063 inhibitor treatment upregulated H9C2 cell viability, downregulated apoptosis, and eliminated the effects of CCAT1 knockdown on DEX-and H/R-treated H9C2 cells (Figure 5(b,c)). Moreover, western blotting showed that the miR-8063 inhibitor reduced the protein levels of Wnt3a, Wnt5a, and β-catenin and partially reversed the effects of CCAT1 knockdown on the activation of the Wnt/β-catenin pathway (Figure 5(d)). These results suggest that miR-8063 interference promotes cells viability, inhibits apoptosis, and inactivates the Wnt/β-catenin pathway, thereby reversing the effects of CCAT1 knockdown on H/R H9C2 cells.

**Figure 5.** Interfering with miR-8063 reverse the effect of knockdown CCAT1 on the viability and apoptosis of H/R H9C2 cells (a). miR-8063 level of H9C2 cells among inhibitor-NC, inhibitor, si-NC, si-CCAT1, si-CCAT1 + inhibitor groups were assayed by qRT-PCR. (b). The cell viability of H9C2 cells in H/R, H/R + DEX, H/R + DEX +si-NC, H/R + DEX +si-CCAT1, H/R + DEX +si-CCAT1 + inhibitor-NC, and H/R + DEX +si-CCAT1 + inhibitor groups was assessed by CCK-8. (c). FITC-PI kit was employed to assess cell apoptosis in H/R, H/R + DEX, H/R + DEX +si-NC, H/R + DEX +si-CCAT1, H/R + DEX +si-CCAT1 + inhibitor-NC, and H/R + DEX +si-CCAT1 + inhibitor groups. (d). Western blotting was utilized to measure Wnt3a, Wnt5a and β-catenin protein levels in H9C2 treated with H/R, H/R + DEX, H/R + DEX +si-NC, H/R + DEX +si-CCAT1, H/R + DEX +si-CCAT1 + inhibitor-NC, and H/R + DEX +si-CCAT1 + inhibitor. H/R, hypoxia/reoxygenation; Dex, dexmedetomidine; si-CCAT1, CCAT1 siRNA; si-NC, negative control of si-CCAT1; inhibitor, miR-8063 inhibitor; inhibitor-NC, negative control of miR-8063 inhibitor. N = 3 for each group.

## Discussion

H9C2 cells were used to establish an H/R injury model, and Dex and CCAT1/miR-8063/Wnt/β-catenin were analyzed to reveal the cardioprotective mechanism induced by Dex preconditioning. We observed that Dex treatment alleviated the decrease in H9C2 cell viability, enhanced the apoptosis, and activated the Wnt/β-catenin pathway induced by H/R. Additionally, the expression levels of CCAT1 were downregulated in H/R H9C2 cells, which was reversed by Dex treatment. Furthermore, CCAT1 knockdown inhibited H/R H9C2 cell viability, promoted apoptosis, and activated the Wnt/β-catenin pathway by upregulating miR-8063 expression.

As a new class of ncRNA molecules, lncRNAs play crucial roles in the development of cardiovascular diseases. For example, overexpression of lncRNA AK006774 reduces the I/R-induced infarct size in vivo and inhibits the apoptosis and oxidative stress in cardiomyocytes after H/R treatment in vitro [26]. Loss of lncRNA 2810403D21Rik/Mirf promotes autophagy, reduces cardiac injury, and improves cardiac function in mice with acute myocardial infarction [27]. Inhibition of the X inactive specific transcript in H9C2 cells and I/R mice leads to apoptosis and autophagy reduction and promotes cell viability [28]. The lncRNA receptor tyrosine kinase like orphan receptor accelerates H/R-induced cardiomyocyte injury [29]. In addition, as an anesthetic that has a regulatory effect on lncRNAs, Dex is often combined with lncRNAs in the study of various diseases [10]. For example, Dex modulates the lncRNA small nucleolar RNA host gene 16 to ameliorate neuronal injury in ischemic stroke and exert neuroprotective effects [30]. Dex downregulates the activation of spinal cord I/R injury in mice and OGD/R-treated primary microglia [31].

Various studies on the roles of CCAT1 and Dex in OGD/R hepatocytes have been reported [17]. This study explored the impact of CCAT1 and Dex on the apoptosis and viability of H/R-treated H9C2 cells. Consistent with previous studies, Dex pretreatment alleviated the H/R-induced decrease in cell viability and increased the apoptosis of H9C2 cells. Similar to its effect in hepatocytes, CCAT1 levels were downregulated in H/R H9C2 cells, and this effect was reversed by Dex. Additionally, CCAT1 knockdown reversed the H/R-mitigating effects of Dex. These data indicate that Dex could attenuate H/R-induced myocardial cell apoptosis by upregulating CCAT1 levels, which provides a basis for Dex-mediated regulation of lncRNA to reduce H/R-induced cardiomyocyte damage.

miRNA, another type of ncRNA, plays an essential role in myocardial injury caused by ischemia and hypoxia. For example, overexpression of miR-129-5p effectively reduces the myocardial infarct size and myocardial apoptosis rate in rats with myocardial I/R damage [32]. miR-374a-5p may have a protective impact on H/R impairment in vitro and cardiac I/R injury in vivo [33]. In this study, we found that miR-8063 levels were upregulated in H/R-induced H9C2 cells due to pretreatment with Dex. Further functional studies showed that the knockdown of miR-8063 promoted cardiomyocyte viability and inhibited their apoptosis. Therefore, Dex may play a protective role by inhibiting the expression of miR-8063.

LncRNAs function as competitive endogenous RNAs (ceRNAs) by sponging specific miRNAs, reducing miRNA abundance and alleviating the inhibition of downstream target genes [34]. The lncRNA–miRNA regulatory network plays essential roles in many diseases. For example, lncRNA XLOC, a ceRNA that targets miR-331-3p and miR-338-3p, promotes tumorigenesis and metastasis in cervical cancer [35]. Silencing of lncRNA growth arrest specific 5 may protect H9C2 cells from hypoxia-induced injury via the sponge action of miR-142-5p [36]. Interestingly, our data suggest that CCAT1 combined with miR-8063 acts as a ceRNA. In addition, functional assays showed that interference with miR-8063 had similar effects on H/R H9C2 cells and reversed H/R deterioration induced by low expression of CCAT1.

The Wnt/β-catenin signaling pathway is involved in many biological processes, such as cell apoptosis, differentiation, and proliferation, and is an important regulator of embryogenesis and physiological growth [37]. Wnt triggers signal transduction cascades mediated by receptors. After binding to receptors, Wnt can activate various outputs in a β-catenin-dependent (typical response) or β-catenin-independent (atypical response) manner [38,39]. Typical and atypical Wnt signals are triggered by different Wnt proteins, which block the degradation of β-catenin in typical reactions. Furthermore, Wnt3a is considered an effective stimulator of the β-catenin-dependent response, while Wnt5a activates the β-catenin-independent signals [40]. An increasing number of studies have focused on the role of the Wnt/β-catenin signaling pathway in H/R-mediated cardiomyocyte injury. For example, Wang et al. [18] found that the Wnt/β-catenin signaling pathway is activated in H/R-induced H9C2 cells, resulting in increased expression levels of Wnt3a, Wnt5a, and β-catenin. Yan et al. [41] Moreover, they found that Dex treatment inhibited the activation of the H9C2 Wnt/β-catenin signaling pathway [18]. The results of this study are consistent with those in the literature, which found that the expression levels of Wnt3a, Wnt5a, and β-catenin in H9C2 were increased after H/R injury, and that the upregulation of these protein levels was partially reversed by Dex treatment. In addition, our study showed that CCAT1 knockdown activated the Wnt/β-catenin signaling pathway, which was inhibited by miR-8063 interference. These result are contrary to the previously reported roles of CCAT1 and miR-8063 in cancer [42,43]. We suspect that this is due to differences in the disease. In summary, our results suggest that the Wnt/β-catenin signaling pathway is involved in Dex-CCAT1/miR-8063-mediated H9C2 anti-H/R damage.

The crosstalk modulation mechanisms among the lncRNA, miRNA, and mRNA play essential roles in the pathophysiology of cardiovascular diseases in response to stress stimuli [44]. We aim on finding the downstream mRNA of CCAT1/miR-8063 and exploring its effect on the function of H/R cardiomyocytes. In addition, in vivo experiments can provide convincing evidence for the protective effect of Dex in the myocardium to prevent H/R impairment. However, various complex physiological processes are always occurring in the body that may be associated with various related mechanisms, and the role of a single lncRNA or miRNA in the body may be limited. In the future, we aim to establish a rat H/R model to study the possible mechanism of Dex in vivo.

## Conclusion

In conclusion, we have demonstrated that Dex exerts significant protective effects against H/R-mediated cardiomyocyte injury. Mechanistically, Dex works by inducing CCAT1 expression in the sponge miR-8063 and inactivating the Wnt/β-catenin signaling pathway. Herein, we revealed the myocardial protection provided by Dex during H/R-mediated H9C2 cell injury and its possible underlying mechanism, offering a novel theoretical basis for the treatment of this injury.

## Data Availability

The datasets used and/or analyzed during the current study are available from the corresponding author on reasonable request.
